# Efficacy and safety of lenvatinib monotreatment and lenvatinib-based combination therapy for patients with unresectable hepatocellular carcinoma: a retrospective, real-world study in China

**DOI:** 10.1186/s12935-021-02200-7

**Published:** 2021-09-18

**Authors:** Yun Zhu, Penghui Sun, Kunyuan Wang, Shuzhe Xiao, Yanling Cheng, Xiangzhao Li, Biao Wang, Jiancong Li, Wenxuan Yu, Yang Cheng

**Affiliations:** 1 Liver Tumor Center, Department of Infectious Diseases and Hepatology Unit, Nanfang Hospital, Southern Medical University, Guangzhou, 510515 Guangdong China; 2 Nanfang PET Center, Nanfang Hospital, Southern Medical University, Guangzhou, 510515 Guangdong China; 3 Digestive Department, Guangzhou Women and Children’s Medical Center, Guangzhou Medical University, Guangzhou, 510623 Guangdong China; 4 Department of Pathology, Nanfang Hospital, Southern Medical University, Guangzhou, 510515 Guangdong China; 5 Department of Hepatobiliary Surgery, Nanfang Hospital, Southern Medical University, Guangzhou, 510515 Guangdong China

**Keywords:** Lenvatinib, Monotreatment, Combination therapy, Hepatocellular carcinoma

## Abstract

**Background:**

Lenvatinib and lenvatinib-based combination treatments are widely used in patients with unresectable hepatocellular carcinoma (uHCC) in clinical practice, but their curative effect and safety need further study in the real world.

**Methods:**

This was a retrospective study involving patients with uHCC receiving lenvatinib monotherapy and lenvatinib-based combination treatment between Nov, 2018 and Sep, 2020 in Nanfang Hospital. Efficacy was evaluated with objective response rate (ORR), disease control rate (DCR), progression-free survival (PFS), time to tumor progression (TTP), and overall survival (OS). Treatment-related adverse events (TRAEs) were recorded and graded. Efficacy and safety of monotherapy and combination therapy were compared. Stratified analysis was performed according to systemic line of treatment and medication regimen for combination therapy.

**Results:**

For lenvatinib monotherapy (n = 39), OS and PFS were 80 weeks and 24.3 weeks, respectively. For combination treatment (n = 72), median OS and PFS were 99 weeks and 45.6 weeks, respectively. OS, PFS, and TTP for patients in the combination treatment cohort were significantly longer compared to those of patients in the monotreatment cohort (OS: P = 0.04, PFS: P = 0.003; TTP, P = 0.005). The incidence of TRAEs could be controlled both in the monotherapy cohort and the combination treatment cohort. In the monotherapy cohort, OS and PFS were significantly decreased in the second-line treatment group compared with the first-line treatment group, while no differences were observed in the combination cohort. The efficacy of triple therapy (lenvatinib plus PD-1 antibody plus TACE or HAIF) was similar to lenvatinib plus PD-1 antibody or lenvatinib plus TACE or HAIF.

**Conclusions:**

Our real-world study showed that lenvatinib monotherapy and lenvatinib-based combination therapy were well tolerated, with encouraging efficacies in patients with uHCC. Lenvatinib-based combination therapy showed a better curative effect compared with lenvatinib single-agent therapy. In patients who have failed first-line TKI treatment, lenvatinib-based combination therapy may be a better choice than lenvatinib single-agent therapy. Lenvatinib-based triple therapy may not have an advantage over dual therapy.

**Supplementary Information:**

The online version contains supplementary material available at 10.1186/s12935-021-02200-7.

## Introduction

Hepatocellular carcinoma (HCC) is a highly malignant tumor associated with high morbidity and mortality and represents a major public health issue. The incidence of HCC ranks 6th among malignant tumors, and the mortality rate ranks 3rd worldwide. In addition, HCC accounts for 4.7% of all cancers, but 8.3% of cancer-related deaths worldwide. It is estimated that over 830,000 people died of HCC globally in 2020 [1, 2].

Tyrosine kinase inhibitors (TKIs) are widely used in advanced unresectable HCC (uHCC). Sorafenib was the first TKI approved for advanced uHCC [3]. Lenvatinib is a novel TKI for the first-line treatment of HCC, which gained approval in 2018. Although lenvatinib has proven to be superior to sorafenib in increasing the overall survival (OS) in patients with HCC in clinical trials, its effect is limited by drug resistance as well as its intolerable side effects [4]. Although several drugs have been approved for the treatment of HCC in recent years, these drugs are not satisfactory owing to their associated toxicities and the rapid development of drug resistance. HCC is a highly heterogeneous tumor and many molecular pathways are involved in the development of drug resistance in HCC cells; therefore, treating HCC patients remains a challenge. There is an urgent need to develop new combination treatment strategies that target different signal pathways [5] .

Recently, there have been several studies exploring the safety and efficacy of combining TKIs and programmed cell death protein-1 (PD-1)-targeted immunotherapy. In addition, combination treatment with a TKI plus local treatment, such as transcatheter arterial chemoembolization (TACE) or hepatic arterial infusion with drug filtration (HAIF), has also been used. A phase 3 clinical trial showed that the addition of HAIF to sorafenib did not significantly improve OS in patients with advanced HCC [6]. Combination therapy with lenvatinib and PD-1-targeted immunotherapy has shown preliminary efficacy in the first-line treatment of HCC. PD-1-targeted immunotherapy, as a checkpoint inhibitor, shows promising efficacy and safety in patients with advanced HCC [7, 8]. However, not all patients show responses to checkpoint inhibitor-based therapy. Additionally, there are many side effects of PD-1 targeted treatment, such as fatigue, rash, decreased appetite, thyroid dysfunction, immune colitis, autoimmune hepatitis, and immune-related pneumonia [7, 9]. Repeated TACE has been an important local therapeutic strategy for HCC; however, there is a potential risk of liver damage or even liver failure associated with this treatment [10]. HAIF has proven to be an effective and safe treatment in advanced HCC and may improve both progression-free survival (PFS) and OS in patients with advanced HCC [11].

Whether combination therapy significantly improves efficacy and whether it increases side effects is a concern of clinicians. However, the beneficial effects and side effects of lenvatinib-based combination treatment in HCC in the real world remain unclear.

In the last three years, a subset of HCC patients in our center were treated with lenvatinib monotherapy, including some who were treated with lenvatinib-based combination treatment,such as lenvatinib plus PD-1 antibody and lenvatinib plus local treatment. We conducted a retrospective study to evaluate the efficacy and side effects of the real-world use of these therapies in patients with HCC.

## Methods

### Study design and patients

This was a retrospective single-center real-world study of patients who received lenvatinib monotherapy or lenvatinib-based combination treatment. Patients treated with lenvatinib (n = 39) or lenvatinib-based combination treatment (n = 72) between Nov, 2018 and Sep, 2020 were enrolled. All patients were pathologically or clinically diagnosed with HCC according to the standards of the American Association for the Study of Liver Diseases (AASLD) [12]. This study was part of a larger trial (observational study of primary liver cancer) which was approved by the Ethics Committee of Nanfang Hospital, Southern Medical University (2020ZX09201017). The study design flow chart is shown in Fig. 1.

**Fig. 1:** Flow chart of study design

### Study treatment

Patients received oral lenvatinib (12 mg/day for bodyweight ≥ 60 kg and 8 mg/day for bodyweight < 60 kg). For treatment with PD-1 antibodies, patients received intravenous toripalimab (240 mg every 3 weeks), camrelizumab (200 mg every 3 weeks), sintilimab (200 mg every 3 weeks), tislelizumab (200 mg every 3 weeks), or pembrolizumab (2 mg/kg every 3 weeks). For TACE or HAIF treatment, patients received TACE / HAIF every one or two months.

### Assessments

Clinical and laboratory data from eligible patients were collected prior to initiation of lenvatinib or lenvatinib combination therapy. Tumor staging was determined according to the Barcelona Clinic Liver Cancer (BCLC) staging system, and included Eastern Cooperative Oncology Group (ECOG) performance status, Child-Pugh score, tumor size, tumor number, vascular invasion, and extrahepatic metastasis. Patient characteristics are shown in Table 1. Tumor evaluation was based on enhanced computed tomography (CT) or magnetic resonance imaging (MRI). Patients underwent baseline contrast CT/MRI and contrast CT/MRI at follow-up every 6–12 weeks. Response evaluation criteria in solid tumors (RECIST) was used to evaluate tumor responses [12, 13]. The specific criteria were as follows: (1) complete response (CR), all target lesions disappeared; (2) partial response (PR), the total diameter of the target lesion was reduced by 30% or more; (3) stable disease (SD), the total diameter of the target lesion was not reduced as classified in PR and not increased as classified for disease progression; (4) progressive disease (PD), the total diameter of the target lesions increased by 20% or more or new lesions appeared. Treatment-related adverse events (TRAEs) were recorded and graded according to the Common Terminology Criteria for Adverse Events (CTCAE) version 5.0.

**Table 1:** Baseline characteristics of patients

	LEN monotherapy (n = 39)	LEN combination (n = 72)	LEN + PD1 (n = 30)	LEN + HAIF/TACE (n = 24)	LEN + PD1 + HAIF/TACE (n = 16)
Age (Median ± SE)	50 ± 13.3	51 ± 11.9	50.5 ± 10.6	55 ± 13.1	50 ± 12.8
Gender (Male/Female)	37/2	66/6	28/2	23/1	13/3
BCLC stage (A/B/C)	6/11/22	11/14/47	5/5/20	3/5/16	3/3/10
HBV infection (Yes/No)	33/6	65/7	28/2	22/2	13/3
AFP (ng/ml) (< 400/> 400)	24/15	33/39	15/15	9/15	8/8
Median follow-up (week)	44.7	45.1	48.9	45.2	36.4
Child-Pugh (A/B)	7/32	7/65	4/26	2/24	16/16

AFP, alpha-fetoprotein; BCLC, Barcelona Clinic Liver Cancer; HAIF, hepatic arterial infusion with drug filtration; HBV, hepatitis B virus; LEN, lenvatinib; PD1, programmed cell death protein-1; TACE, transcatheter arterial chemoembolization

### Statistics

Comparisons of the efficacy of lenvatinib and different PD-1 antibodies were not conducted due to the small sample size of each group after grouping. The primary efficacy endpoint was OS, which was compared between the lenvatinib monotherapy group and the combination treatment group. The secondary endpoints were PFS and time to progression (TTP) in the lenvatinib monotherapy group and combination group. Exploratory analyses were conducted to evaluate treatment efficacy in subgroups of patients who had received different numbers of lines of prior systemic treatment and different kinds of combination therapy.

OS was defined as the time from start of indicated treatment to death. PFS was defined as the time between initiation of indicated treatment to tumor progression or death. TTP was defined as duration from indicated treatment to tumor progression. The objective response rate (ORR) was defined as the proportion of patients with CR or PR after treatment of the total number of evaluable cases. Disease control rate (DCR) was defined as the number of remission and stable cases after treatment as the percentage of the total evaluable cases. Survival analysis was conducted using the Kaplan-Meier method and the log-rank test was used to evaluate the statistical significance of inter-group differences in survival. All statistical analyses were performed using SPSS. P < 0.05 was considered significant.

## Results

### Clinical course of patients

A total of 111 patients who had at least one imaging follow-up and were available for radiological assessment of tumor response between Nov, 2018 and Sep, 2020 were enrolled. Patients not available for tumor response assessment, lost to follow-up, or who died before the first radiological evaluation were excluded. Baseline characteristics of patients are summarized in Table 1. In total, 39 patients received lenvatinib monotherapy during the study period and 72 patients received lenvatinib-based combination treatment. Of the 72 patients who received lenvatinib-based combination treatment, 30 patients received lenvatinib and anti-PD-1 antibodies, 24 received lenvatinib with local treatment (TACE or HAIF), and 16 received triple therapy with lenvatinib plus local treatment (TACE or HAIF) and anti-PD-1 antibodies. One patient received lenvatinib plus microwave ablation. And one patient received lenvatinib plus microwave ablation and local radiotherapy.

Treatments received prior to initiation of lenvatinib therapy are shown in Table 2. Seventeen patients (15.3%) had BCLC A stage disease, 25 patients (22.5%) had BCLC B stage, and 69 patients (62.2%) had BCLC C stage. The mean treatment time of lenvatinib monotherapy was 5.9 months, and the mean treatment time of combination treatment was 8.2 months. The median follow-up period was 44.7 weeks for patients who received lenvatinib monotherapy and 45.0 weeks for patients who received combination treatment.

**Table 2:** Treatment prior to lenvatinib therapy

	LEN monotherapy	LEN combination
First-line treatment	27/69%	62/86%
Second-line treatment	12/31%	8/11%
Sorafenib	12/31%	3/4%
Apatinib	0	3/4%
PD-1 antibody	0	2/3%
Third-line treatment	0	2/3%

Data are presented as n/%

LEN, lenvatinib; PD-1, programmed cell death protein-1

At data cut-off (Feb 2021), 10 (25.6%) and 38 (52.8%) patients were still receiving lenvatinib monotherapy and combination treatment, respectively. Discontinuation of lenvatinib or combination therapy was mainly due to disease progression.

### Efficacy

In the lenvatinib monotherapy group, no patient achieved a CR, 6 (15%) participants achieved a PR, and 21 (54%) individuals had SD. The ORR and DCR for lenvatinib monotherapy were 15 and 69%, respectively (Table 3). Median OS was 80 (95% CI 68–92) weeks, median PFS was 24.3 weeks, and median TTP was 24.3 weeks (Fig. 2).

**Table 3:** Efficacy of lenvatinib in patients with uHCC

	LEN monotherapy (n = 39)	LEN combination (n = 72)	LEN + PD1 (n = 30)	LEN + HAIF/TACE (n = 24)	LEN + PD1 + HAIF/TACE (n = 16)
CR	0	2/3%	1/3%	0	0
PR	6/15%	19/26%	10/33%	7/29%	2/13%
SD	21/54%	42/58%	12/40%	17/71%	12/75%
ORR	15%	29%	36%	29%	13%
DCR	69%	87%	76%	100%	88%

Data are presented as n/%

LEN, lenvatinib; PD-1, programmed cell death protein-1 targeted immunotherapy; HAIF, hepatic arterial infusion with drug filtration; TACE, transcatheter arterial chemoembolization; CR, complete response; ORR, objective response rate; DCR, disease control rate; PR, partial response; SD, stable disease

**Fig. 2:** Kaplan–Meier analysis of overall survival (**A**), progression-free survival (**B**), and time to progression (**C**) in patients receiving lenvatinib monotreatment and lenvatinib-based combination treatment

For patients receiving combination treatment, 3%, 26%, and 58% had a CR, PR, and SD, respectively. The ORR and DCR were 29 and 87%, respectively (Table 3). Median OS was 99 weeks, median PFS was 45.6 weeks, and median TTP was 46.3 weeks for the lenvatinib combination group (Fig. 2).

Survival analysis showed that OS, PFS, and TTP for patients in the combination treatment cohort were all significantly longer compared to that of patients in the monotreatment cohort (OS: P = 0.04, PFS: P = 0.003; TTP, P = 0.005) (Fig. 2). Representative images from patients treated with lenvatinib monotherapy and combination therapy before and after treatment are shown in Fig. 3.

**Fig. 3:** Representative images of liver tumor size in patients before and after lenvatinib treatment. **A** A CT image of a male patient before lenvatinib monotreatment (left) and 23 months after lenvatinib treatment (right). **B** A CT image of a female patient before treatment (left) and 4 months after lenvatinib + PD1 + HAIF treatment (right)

### Safety

In total, 37 (94.9%) patients in the lenvatinib monotherapy group experienced at least one TRAE. The most common adverse events with lenvatinib monotherapy were elevated transaminase (n = 18; 46.2%), anemia (n = 13; 33.3%), proteinuria (n = 12; 30.85%), diarrhea (n = 7; 18.0%), and fatigue (n = 7; 18.0%). Grade 3 or higher adverse events occurred in 28.2% of patients in the lenvatinib monotherapy group (Table 4). A dose delay due to adverse events was required in 10 (27.0%) patients treated with lenvatinib monotherapy. Fatal adverse events related to lenvatinib treatment occurred in 1 patient (2.6%) who had hepatic failure.

**Table 4:** Treatment-related adverse events in HCC patients with Lenvatinib monotherapy

Adverse event	Any grade	Grade I–II	Grade III–V
Any adverse event	37/94.9%	26/66.7%	11/28.2%
Rash	2/5.1%	2/5.1%	0/0.00%
Diarrhea	7/18.0%	6/15.4%	1/2.6%
Anemia	13/33.3%	10/25.6%	3/7.7%
Elevated transaminase	18/46.2%	9/23.1%	9/23.1%
Hypertension	3/7.7%	3/7.7%	0/0.00%
Leukopenia	4/10.3%	4/10.3%	0/0.00%
Hypothyroidism	6/15.4%	6/15.4%	0/0.00%
Bleeding	6/15.4%	6/15.38%	0/0.00%
Proteinuria	12/30.8%	11/28.2%	1/2.6%
Fever	1/2.6%	1/2.6%	0/0.00%
Fatigue	7/18.0%	7/18.0%	0/0.00%
Hand-foot skin reaction	6/15.4%	6/15.4%	0/0.00%
Dysphonia	1/2.6%	1/2.6%	0/0.00%
Decreased appetite	3/7.7%	3/7.7%	0/0.00%
Vomitting	1/2.6%	1/2.6%	0/0.00%

Data are presented as n/%

67 (93.1%) patients in the combination treatment group experienced at least one TRAE. The most common adverse events in the lenvatinib combination therapy group were elevated transaminase (n = 28; 38.9%), proteinuria (n = 25, 34.7%), anemia (n = 23; 31.9%), leukopenia (n = 16; 22.2%), diarrhea (n = 13; 18.1%), thyroid dysfunction (n = 13, 18.1%), and hypertension (n = 11; 15.3%) (Table 5). Observed grade 3 or higher adverse events occurred in 23.6% of patients in the combination treatment group. A dose delay due to adverse events was required in 18 (25.0%) patients in the combination treatment group (Table 5). Fatal adverse events related to combination treatment occurred in 1 patient (1.4%), who had intestinal hemorrhage.

**Table 5:** Treatment-related adverse events in HCC patients with Lenvatinib based combination treatment

Adverse Event	Any Grade	Grade I–II	Grade III–V
Any adverse event	68/94.4%	49/68.5%	19/26.3%
Rash	7/9.7%	7/9.7%	0/0.00%
Diarrhea	13/18.1%	10/13.9%	3/4.2%
Anemia	23/31.9%	16/22.2%	7/9.7%
Elevate transaminase	28/38.9%	21/29.2%	7/9.7%
Hypertension	11/15.3%	8/11.1%	3/4.2%
Leukopenia	16/22.2%	12/16.7%	4/5.6%
Thyroid dysfunction	13/18.1%	13/18.1%	0/0.00%
Constipation	4/5.6%	4/5.6%	0/0.00%
Bleeding	8/11.1%	8/11.1%	0/0.00%
Vision loss	1/1.4%	1/1.4%	0/0.00%
Proteinuria	25/34.7%	25/34.7%	0/0.00%
Fever	2/2.8%	2/2.8%	0/0.00%
Fatigue	9/12.5%	9/12.5%	0/0.00%
Hand-foot skin reaction	10/13.9%	10/13.9%	0/0.00%
Decreased appetite	4/5.6%	4/5.6%	0/0.00%
Vomitting	3/4.2%	3/4.2%	0/0.00%
Bloody stools	1/1.4%	1/1.4%	0/0.00%

Data are presented as n/%

In terms of safety, the proportions of patients who developed any grade or high grade adverse events were similar between lenvatinib monotherapy and lenvatinib combination therapy.

### Efficacy according to line of systemic treatment

In the lenvatinib monotreatment group, 27 patients (69%) received lenvatinib as the first-line systemic treatment, and 12 patients (31%) received it as a second-line systemic treatment. ORR and DCR for first-line treatment vs. second-line treatment were 19% vs. 8% and 63% vs. 83%, respectively (Table 6). Survival analysis showed that OS and PFS were significantly lower in the second-line systemic treatment subgroup compared with the first-line systemic treatment subgroup (Fig. 4A, B).

**Table 6:** Efficacy of first-line treatment and second-line treatment in lenvatinib monotreatment group

LEN (n = 39)	First-line treatment (n = 27)	Second-line treatment (n = 12)
CR	0	0
PR	5	1
SD	12	9
PD	10	2
ORR	19%	8%
DCR	63%	83%

LEN, lenvatinib; CR, complete response; PR, partial response; SD, stable disease; PD, progressive disease; ORR, objective response rate; DCR, disease control rate

**Fig. 4:** Subgroup analysis according to line of systemic treatment. Kaplan–Meier analysis of overall survival (**A**) and progression-free survival (**B**) in patients receiving lenvatinib monotreatment. Kaplan–Meier analysis of overall survival (**C**) and progression-free survival (**D**) in patients receiving combination treatment

In the lenvatinib combination treatment group, 62 patients (86%) received lenvatinib as first-line treatment, 8 patients (11%) in second-line, and 2 patients (3%) in third-line. As there was a low number of patients who received lenvatinib combination therapy in third-line, we grouped patients into a first-line treatment group and a non-first-line treatment group (second- or third-line treatment). ORR and DCR for first-line treatment vs. non-first-line treatment were 32% vs. 10 and 87% vs. 90%, respectively (Tables 6, 7). There was no significant difference in OS or PFS between the first-line treatment subgroup and non-first-line treatment subgroup (Fig. 4C, D).

**Table 7:** Efficacy of first-line treatment and non-first line treatment in lenvatinib combination treatment group

LEN combination treatment	First line treatment (n = 62)	Second line treatment (n = 8)	Third-line treatment (n = 2)	Non-first line treatment (n = 10)
CR	1	0	1	1
PR	19	0	0	0
SD	34	8	0	8
PD	8	0	1	1
ORR	32%	0%	50%	10%
DCR	87%	100%	50%	90%

CR, complete response; DCR, disease control rate; LEN, lenvatinib; ORR, objective response rate; PD, progressive disease; PR, partial response; SD, stable disease

### Efficacy subgroup analysis by type of combination therapy

In the lenvatinib plus anti-PD-1 antibody group, 1 (3%) and 10 (33%) patients achieved a CR or PR, respectively and 12 (40%) patients had SD. The ORR and DCR for the lenvatinib plus anti-PD-1 antibody cohort were 36 and 76%, respectively (Table 3). In the lenvatinib plus TACE/HAIF-treated patients, no patients achieved a CR, and 7 (29%) and 17 (71%) participants achieved a PR and SD, respectively. The ORR and DCR for the lenvatinib plus TACE/HAIF cohort were 29 and 100%, respectively (Table 2). In the lenvatinib plus TACE/HAIF and anti-PD-1 antibody cohort, no participants achieved a CR, and 2 (13%) and 12 (75%) patients showed a PR and SD, respectively. The ORR and DCR for this cohort were 13 and 88%, respectively (Table 2).

Median OS for the lenvatinib plus anti-PD-1 antibody cohort was 88.7 weeks and median PFS was 43.6 weeks. Median PFS for the lenvatinib plus TACE/HAIF cohort was 47.7 weeks. Median OS for the lenvatinib plus TACE/HAIF cohort and lenvatinib plus TACE/HAIF and anti-PD-1 cohort has not been reached. Median PFS for the lenvatinib plus TACE/HAIF and anti-PD-1 cohort has also not been reached. The results of subgroup analysis showed that there was no significant difference in OS and PFS between the different combination treatment groups (Fig. 5).

**Fig. 5:** Subgroup analysis of the combination therapy group according to treatment. Kaplan–Meier analysis of overall survival (**A**) and progression-free survival (**B**) in patients receiving lenvatinib plus PD-1 antibodies, lenvatinib plus TACE/HAIF, or lenvatinib plus PD-1 antibodies and TACE/HAIF

Moreover, we conducted a subgroup analysis in patients who received lenvatinib and local treatment according to the local treatment method. As shown in Fig. 6, there was no significant difference in OS and PFS between patients receiving HAIF and TACE.

**Fig. 6:** Subgroup analysis of combination therapy according to local treatment. Kaplan–Meier analysis of overall survival (**A**) and progression-free survival (**B**) in patients receiving monotreatment

## Discussion

Hepatitis B virus (HBV) infection is the major cause of liver cirrhosis and HCC in China [14]. HBV infections may develop into HCC due to genetic mutations induced by HBV [15]. Over 80% of HCC patients in China have an HBV infection. Our cohort was representative of this and 89% of patients had an HBV infection. To the best of our knowledge, this is the first real-world study evaluating lenvatinib and lenvatinib combination treatment in patients with HBV-related HCC.

In our single-center, real-world study, Chinese HCC patients who received lenvatinib monotherapy had an OS of 18.7 months vs. 13.6 months in the Phase III REFLECT trial, the PFS was 5.6 months vs. 7.3 months in the REFLECT trial, and the TTP was 5.6 months vs. 7.4 months in the REFLECT trial [4]. TRAEs occurred in 94.9% of the patients in our study vs. 98.7% in the REFLECT trial. The most common TRAEs for lenvatinib treatment in our study were elevated transaminase (46.2%), anemia (33.3%), proteinuria (30.85%), diarrhea (18.0%), and fatigue (18.0%). The side effect spectrum observed in the present study was slightly different from that in the REFLECT trial. For example, the rate of grade 3 or higher TRAEs was much lower in our study compared with the REFLECT trial (28.2% vs. 75%). The dose interruption rate was also lower than that in the REFLECT trial (27% vs. 40%). In summary, our study supports the treatment effect and safety of lenvatinib monotherapy reported in the REFLECT study.

In this study, we conducted a stratified analysis based on patient’s previous treatment, and the results suggest that patients receiving lenvatinib treatment in first-line had significantly longer OS and PFS than those who were treated with lenvatinib in second line. To our knowledge, this is the first study comparing first-line versus second-line lenvatinib treatment. Our results suggest that lenvatinib is more advantageous when used as a first-line treatment than as a second-line treatment.

Combination treatment strategies that combine molecular targeted therapies with PD-1-targeted immunotherapies are currently being explored in patients with uHCC. These combination therapy approaches are extremely promising because combining the two drugs produces not just an additive effect, but rather a synergistic effect against the immunosuppressive tumor microenvironment [16, 17]. In our study, lenvatinib-based combination treatment led to a higher ORR and DCR, as well as longer OS and PFS versus lenvatinib monotherapy. This finding suggests that combination therapy had better efficacy than monotherapy, which is in-line with the conclusions of the existing literature. Furthermore, in our study, the safety of lenvatinib combination treatment was similar to lenvatinib monotherapy, with comparable incidences of TRAEs and severe TRAEs in the two groups.

There have been a number of recent phase Ib/II clinical studies exploring the treatment effects of an anti-PD-1 antibody combined with lenvatinib for HCC patients. A phase I clinical study of lenvatinib plus pembrolizumab, which enrolled 13 HCC patients with BCLC stage B/C disease, showed that 46%, 46%, and 92% of patients achieved a PR, SD, and DCR, respectively. TRAEs occurred in 94% of patients in this study, and the most common TRAEs were decreased appetite and hypertension [18]. In our cohort of 30 HCC patients receiving lenvatinib plus anti-PD-1 antibodies, 33% achieved a PR, 40% achieved SD, and the DCR was 76%. TRAEs occurred in 96.7% of the patients, and grade 3 TRAEs occurred in 26.7%; there were no grade 4 or 5 TRAEs. Similar to the results of the above phase I clinical study, our study suggests that combined lenvatinib and anti-PD-1 antibody therapy achieved a remarkable antitumor effect and controllable side effects.

Clinical studies of new combination therapies for HCC, which combine lenvatinib with TACE/HAIC or lenvatinib plus pembrolizumab with TACE are currently recruiting study participants. However, no preliminary research results have been reported yet. Our research shows that lenvatinib combined with TACE/HAIC yielded a remarkable antitumor effect with an ORR of 29% and DCR of 100%. Moreover, we noticed that in the subgroup analysis of lenvatinib combination treatment, the efficacy of triple therapy (lenvatinib plus anti-PD-1 antibody plus TACE or HAIF) was similar to lenvatinib plus anti-PD-1 antibodies or lenvatinib plus TACE or HAIF. This suggests that triple therapy may not be more advantageous than dual therapy. We plan to conduct a prospective study to compare the efficacy of lenvatinib-based triple therapy and dual therapy to further verify this conclusion.

A prospective, non-randomized, phase II study showed that HAIF yielded significantly better treatment responses than TACE for patients with massive uHCC [19]. In our study, the effect of lenvatinib combined with TACE was similar to that of lenvatinib combined HAIF. This may be due to the small sample size in each group. We will further expand the sample size to verify this conclusion.

There are two main limitations to our study, in addition to the inherent biases present in real-world observational studies. Firstly, this study was retrospectively designed which has inherent limitations including selection bias. Secondly, the sample size was relatively small, particularly for the subgroup analysis, which may have resulted in a reduced statistical power and a risk of bias.

In conclusion, our real-world study showed that lenvatinib monotherapy and lenvatinib-based combination therapy were well tolerated with encouraging efficacy in patients with uHCC. Compared with monotherapy, combination therapy showed a better curative effect without significantly increasing the incidence of adverse reactions. In patients who failed a first-line TKI treatment, lenvatinib-based combination therapy may be a better choice than lenvatinib single-agent therapy. Lenvatinib-based triple therapy may not be more advantageous than dual therapy.

## Supplementary Information

**Additional file 1.** Original data.

## Data Availability

The raw data required to reproduce these findings cannot be shared at this time as the data also form part of an ongoing study.
